The article "Omadacycline Efficacy against Streptococcus Agalactiae Isolated in China: Correlation between Resistance and Virulence Gene and Biofilm Formation" was published in 2022. Journal: Comput Intell Neurosci.

# Omadacycline Efficacy against *Streptococcus Agalactiae* Isolated in China: Correlation between Resistance and Virulence Gene and Biofilm Formation

**DOI:** 10.1155/2022/7636983

**Published:** 2022-04-25

**Authors:** Guiqiu Li, Ying Wei, Yan Guo, Hui Gong, Jie Lian, Guangjian Xu, Bing Bai, Zhijian Yu, Qiwen Deng

**Affiliations:** ^1^Laboratory Medicine Center, Huazhong University of Science and Technology Union Shenzhen Hospital and the 6th Affiliated Hospital of Shenzhen University, Guangdong Shenzhen 518082, China; ^2^Heilongjiang Medical Service Management Evaluation Center, Heilongjiang, Haerbin 150081, China

## Abstract

This study aimed to evaluate the activity, resistance, clonality of MIC distribution, and the correlation between virulence and resistance genes and biofilm formation of omadacycline (OMC) in clinics for *Streptococcus agalactiae* isolates from China. 162 isolates were collected retrospectively in China. The *S. agalactiae* were collected from the body's cervical secretions, wound secretions, ear swabs, secretions, semen, venous blood, cerebrospinal fluid, pee, etc. The MIC of OMC against *S. agalactiae* was determined by broth microdilution. The inhibition zone diameters of OMC and other common antibiotics were measured using filter paper. D-test was performed to determine the phenotype of cross resistance between erythromycin and clindamycin. In Multilocus sequence typing (MLST), some commonly-detected resistance genes and virulence gene of these *S. agalactiae* isolates were investigated using polymerase chain reaction (PCR). Biofilms were detected by crystal violet staining. Our data demonstrated the correalation of the biofilm formation and OMA antimicrobial susceptibility of S.agalactiae clinical isolates with the carrier of virulence gene scpB. Conclusively, OMC exhibits the robust antimcirobial activity against clinical S. agalactiae isolates from China compared with DOX or MIN, and the carrier of the virulence gene scpB might correlate with the biofilm formation in OMC-resistant *S. agalactiae*.

## 1. Introduction

*S. agalactiae* belongs to group B *Streptococcus* (GBS) [1, 2]. *S. agalactiae* is a gram-positive cocci that is microscopically examined for long-chain or long-chain chain arrangement. There are 10 serotypes in III, IV, V, VI, VII, VIII, and IX [3, 4]. *S. agalactiae* is ubiquitous in the natural environment and can reside in the human reproductive tract and digestive tract [5], which is the main pathogenic bacteria in humans and animals [6]. *S. agalactiae* is the most important pathogenic bacteria causing mastitis in dairy cows [7]. *S. agalactiae* has strong infectivity isolated in the primary culture area of tilapia [8]. Human-derived *S. agalactiae* can cause morbidity or even death in newborns, pregnant women, the elderly, and immunocompromised people [9]. Human-derived *S. agalactiae* mainly causes endometritis in women and meningitis, sepsis, and pneumonia in infants and young children. Among them, the infection rate in pregnant women is higher. Previous studies have reported that about 15% to 40% of adult women carry or are infected with *S. agalactiae*, and 25% pass it on to babies; among them, 2% of infants show clinical symptoms, and the mortality rate can be up to 50%. Most of the surviving children have permanent neurological sequelae. The invasive neonatal infections caused by them have caused widespread concern worldwide [10–13].

The article "Omadacycline Efficacy against Streptococcus Agalactiae Isolated in China: Correlation between Resistance and Virulence Gene and Biofilm Formation" was published in 2022. Journal: Comput Intell Neurosci.

Recently, with the widespread use of antibiotics, multidrug resistance has become more serious problem in *S. aglactiae*. High frequence of antibiotics resistance toward erythromycin, clindamycin, and tetracycline has been widely reported in S. aglactiae clinical isolates from China [14–16]. Over 30% of clinical isolates of *S. agalactiae* in Italy has shown the antibiotic resistance toward clindamycin and erythromycin [16–20]. Biofilm formation often enhances the bacterial resistance. Moreover, the bacteria resistance is often correlated with the virulence factors and resistance genes [20–23]. However, the relationship between resistant gene and biofilm formation of *S. agalactiae* is rarely reported.

Omadacycline (OMC) is a new first-in-class aminomethylcycline antibiotic against a widespectrum of gram-positive and negative aerobic bacteria, atypical and anaerobic pathogens [24–27]. OMC has been approved by FDA for the treatment of acute skin and soft tissue infections and community-acquired pneumonia [28, 29]. Susceptibility testing results in limited studies have demonstated the antimcirobial activity of OMC against a wide range of multidrug resistant gram-positive pathogens, such as methicillin-resistant *S. aureus*, vancomycin (Van)-resistant enterococci [8–11]. However, the the antimcirobial susceptibility of OMC against clinical isolates of *S. agalactiae* from China remains elusive [30]. The relationship of OMC susceptitibility with the distribution of these resistance and virulence factors in *S. agalactiae* remains unclear [26].

OMC belongs to a member of the tetracycline (Tet) class. Several tet-specific resistance genes, including tet (M), tet (K), tet (L), tet (A), tet (O), and tet (B), have been found to be correlated with the antibiotic resistance [25–30]. The antimicrobial activity of OMC against *S. agalactiae* harboring Tet-specific resistance genes in vitro has not been clarified yet [28–30].

The article "Omadacycline Efficacy against Streptococcus Agalactiae Isolated in China: Correlation between Resistance and Virulence Gene and Biofilm Formation" was published in 2022. Journal: Comput Intell Neurosci.

This study aimed to evaluate the antimicrobial activity of OMC and its relationship with the resistance factors, virulence factors, and clonality of *S. agalactiae* from China. Here, the MIC of OMC against *S. agalactiae* by both microdilution were examined. The MLST, virulence factors, and resistance gene of these isolates were investigated by PCR. Biofilms were detected by crystal violet staining. The correlation between resistance and resistance genes and biofilm formation was calculated and observed.

## 2. Materials and Methods

### 2.1. Bacterial Isolates, Culture, and Chemicals

162 nonduplicate clinical *S. agalactiae* strains were collected from patients at Shenzhen Nanshan People's Hospital as our previous report [5]. Bacterial species were identified by standard methods using a VITEK 2 compact system (Biomérieux, Marcy l'Etoile, France). The *S. agalactiae* strains were cultured in 5% calf serum in TSB broth medium in a 37°C constant temperature shaker for 18–24 h and then removed. The OMC was purchased from MedChem Express (Princeton, NJ). Thetigecycline, doxycycline, minocycline, eravacylcine, radezolind, erythromycin, solithromycin, telavancin, cefprozil, tetracycline, clindamycin, chloramphenicol, and levofloxacin were purchased from Aladdin (Shanghai, China).

### 2.2. Antibiotic Susceptibility Testing

Antimicrobial susceptibility of OMC and several common antibiotics, including tigecycline, doxycycline, minocycline, eravacylcine, radezolind, erythromycin, solithromycin, telavancin, cefprozil, tetracycline, clindamycin, chloramphenicol, and levofloxacin, were examined by broth microdilution using the VITEK 2 compact system as before. The MICs and inhibition zone diameter of antibiotics was determined, respectively, according to the 2020 Clinical and Laboratory Standards Institute (CLSI) guidelines. The MIC breakpoints of omadacycline, tigecycline, doxycycline, minocycline, eravacylcine, radezolind, erythromycin, solithromycin, telavancin, cefprozil, tetracycline, clindamycin, chloramphenicol, and levofloxacin were selected from the 2020 CLSI. The MIC breakpoint of OMC is ≤ 0.25 mg/L as susceptible; 0.5 mg/L as intermediate; and ≥1 mg/L as resistant, which were selected following previous literature.

### 2.3. D-Test for Detecting the Incidence of Erythromycin Resistance to Inductively Clindamycin

We spread the *S. agalactiae* with a concentration of 0.5 McLaren's turbidity tube on the MH agar plate, applied erythromycin and clindamycin paper at 15 mm intervals, and placed in a constant temperature incubator at 35°C for 16–18 hours. When the bacteriostatic ring of clindamycin paper seemed to be a capital “D”, it was judged as a “D” test positive, indicating that erythromycin had induced clindamycin resistance.

The article "Omadacycline Efficacy against Streptococcus Agalactiae Isolated in China: Correlation between Resistance and Virulence Gene and Biofilm Formation" was published in 2022. Journal: Comput Intell Neurosci.

### 2.4. qRT-PCR Analysis

qRT-PCR was used to analyze MLST and detect resistance and virulence genes. Total bacterial RNA was extracted from *S. agalactiae* isolates and reverse transcribed into cDNA. The Beijing Liuhe Huada Gene Company synthesized the primers for resistance and virulence genes. The cultures of the bacterial strains grew for 4 h at 37°C for overnight. Following the manufacturer instructions, we extract the genomic DNA of the strain, and store at −20°C for future use.

The system for amplification of qRT-PCR (50 *μ*L): Dream Taq Green PCR Master Mix (2×) 25 *μ*L, forward primers 1 *μ*L and reverse primers 1 *μ*L, DNA 2 *μ*L, added ddH_2_O to make up to 50 *μ*L.

qRT-PCR reaction conditions: predenaturation at 95°C for 3 min; denaturation at 95°C for 30 s, annealing at 52°C for 30 s, extension at 72°C for 1 min, 30 cycles; and 72°C for 10 min.

The RNA was submitted to qRT-PCR after adding the qRT-PCR Master Mix (Thermo Fisher Scientific, Waltham, MA, USA). The products of qRT-PCR were stored at 4°C. The *recA* served as an internal control gene. The threshold cycle (Ct) numbers were analyzed using the 2−ΔΔCt method. The qRT-PCR reaction products were electrophoresed on a 1% agarose gel and judged and analyzed according to the presence or absence of positive amplification products and the length of the target gene fragment. All qRT-PCRs were conducted in triplicate.

### 2.5. Crystal Violet Staining for Investigating Resistance and Virulence Gene of the Isolates Detection of Biofilms

After bacteria grew overnight in TSB medium, 200 and TSBG medium were diluted with 0.5% glucose. 200 *μ*L per well was added to 96-well polystyrene microplates with 3 replicate wells, 37°C incubated at room temperature for 24 hours at static temperature. Next, we blotted the pores and rinsed them with PBS 3 times, fixed them with methanol for 15 minutes, stained them with 0.5% crystal violet for 10 minutes, and rinsed them with distilled water. We added 4 : 1 confluence solution of absolute ethanol and acetone, mixed evenly, and tested under OD570 photometry in the end. OG1RF and CHS787 were used as the quality control strains. The interpretation of the biofilm's OD value varies from 0.05 to 3.5 in 96 microwells after staining. Biofilm phenotype classification was based on the method of others, strong positive (OD570 > 2), moderate (OD 570, 1–2), or weak (0.5 < OD570 < 1).

### 2.6. Statistical Analysis

The data were analyzed using a *t*-test by SPSS software. *P* < 0.05 was considered statistically significant.

## 3. Results and Discussion

### 3.1. Antimicrobial Activity and Resistance Analysis of OMC against *S. agalactiae* Isolates Clinical *in Vitro*

The clinical *S. agalactiae* strains were isolated from various infective sample sources, including cervical secretions, wound secretions, ear swab, secretions, semen, venous blood, cerebrospinal fluid, pee, urethral discharge, pus, umbilical secretions, wound secretions, reproductive tract secretions, sputum, gastric juice, throat swab, eye secretions, and amniotic fluid (Figure 1). The MIC and resistance rate of those isolates against antibiotics were obtained (Table 1), and OMC showed *in vitro* resistance against *S. agalactiae*. OMC had robust antimicrobial activity against *S. agalactiae in vitro*, but the clinical *S. agalactiae* isolates exhibited a high-proportion resistance rate to minocycline, erythromycin, solithromycin, and clindamycin. The range of OMC MIC values against *S. agalactiae* was 0.25–1.0 mg/L. The incidence of erythromycin resistance to inductively induced clindamycin against *S. agalactiae* was 90.74% (Table 2), indicating that the incidence of inducing clindamycin resistance was high. The distribution of TET-specific resistance genes in clinical *S. agalactiae* isolates is shown in Figure 2. Our results suggest that the presence of tet (M), tet (O), tet (K), tet (M), and tet (O) genes did not affect OMC sensitivity in *S. agalactiae*.

The article "Omadacycline Efficacy against Streptococcus Agalactiae Isolated in China: Correlation between Resistance and Virulence Gene and Biofilm Formation" was published in 2022. Journal: Comput Intell Neurosci.

### 3.2. Clonality of OMC MIC Distribution

Twenty-one STs were identified among the isolated *S. agalactiae*. The predominant STs were ST10 (32/162; 19.7%) and ST17 (20/162; 12.3%). A new type has been detected. Moreover, 18.8% of ST10 strains and 25.0% of ST17 strains had an OMC MIC level of 1 mg/L, showing clonal clustering toward the ST17 genotype (Table 3).

### 3.3. Formation Characteristics of OMC-Resistant *S. Agalactiae*

The 96-well plate readings after crystal violet staining ranged from 0.13 to 3.10. The median values of the OG1RF strain and the CHS787 control strain OD570 were 1.09 and 1.42, respectively. Among the *S. agalactiae* isolates tested, most of the *S. agalactiae* biofilms showed weak positive and above. Among the strains formed by these biofilms, the weak biofilm phenotypes differed from the medium biofilm phenotypes and the strong. The number of strains in the biofilm phenotype was similar.

### 3.4. The Correlation between Virulence and Resistance Gene and Biofilm Formation

PCR test results suggested that the OMC-resistant *S. agalactiae* resistance-positive genes ermB, ermC, OptrA, msrB, mefAE, tetM, tetO, and tetK were detected, but no ermA, cfr, cfrB, and msrA gene-positive strains were detected (Table 4). The relationship between drug genes and biofilm formation still needs further examination. Statistical analysis showed no significant correlation between genes and biofilm formation (*P* > 0.05). 136 strains of *S. agalactiae* resistant to OMC, analysis of PCR amplified virulence genes showed that bac, bca, fbsA, fbsB, cfb, hylB, Imb, cylE, cpsA, rib, cpsIII, PI-1, PI-2a, and PI-2b positive *S. agalactiae* strains were not statistically correlated with biofilm formation (*P* > 0.05), while the scpB gene was just the opposite of current results, and it was correlated with biofilm formation by statistical analysis (*P* < 0.05) (Table 5).

The article "Omadacycline Efficacy against Streptococcus Agalactiae Isolated in China: Correlation between Resistance and Virulence Gene and Biofilm Formation" was published in 2022. Journal: Comput Intell Neurosci.

## 4. Conclusion

In this study, OMC exhibited robust activity resistance *in vitro* against *S. agalactiae*, and the clinical *S. agalactiae* isolates exhibited a high resistance rate against minocycline, erythromycin, solithromycin, and clindamycin. The main STs observed were ST10 and ST17. The data indicated the clonality of *S. agalactiae* with clustering of the 1 mg/L OMC MIC in the ST17 genotype. The incidence of erythromycin resistance to inductively clindamycin against *S. agalactiae* was higher. Therefore, the clinical microbiology laboratory must strengthen the detection of the *S. agalactiae* D-test, which is resistant to erythromycin and sensitive to clindamycin, to guide the rational clinical use.

The OMC resistance genes ermA, rmB [31], ermC, OptrA, msrB, mefAE, cfr, cfrB, msrA, tetM, tetO, and tetK did not show a significant correlation with biofilm formation. Analysis of PCR amplified virulence genes showed that bac, bca, fbsA, fbsB, cfb, hylB, Imb, cylE, cpsA, rib, cpsIII, PI-1, PI-2a, and PI-2b positive *S. agalactiae* strains have no significant correlation with biofilm formation by statistical analysis (*P* > 0.05) [32–35] whereas the scpB gene was just the opposite to the current result, and it was correlated with biofilm formation by statistical analysis (*P* < 0.05).

To sum up, OMC exhibited robust activity and *in vitro* resistance against *S. agalactiae* isolates, and OMC MIC with 1 mg/L showed ST17 clonality clustering. The incidence of erythromycin resistance to inductively clindamycin against *S. agalactiae* was high [36–38]. The detection of the D-test for *S. agalactiae* must be strengthened in clinics because of its resistance. Biofilm formation ability and OMC resistance genes ermB, ermC, OptrA, msrB, mefAE, tetM, tetO, tetK, ermA, cfr, cfrB, msrA, and virulence genes bca, bac, fbsA, fbsB, cfb, hylB, Imb, cylE, cpsA, rib, cpsIII, PI-1, PI-2a, and PI-2b showed no significant correlation. ScpB was significantly associated with biofilm formation of *S. agalactiae* and OMC-resistant.

## Figures and Tables

**Figure 1:** The clinical *S. agalactiae* strains were isolated from various infective sample sources from 2018 to 2019.

The article "Omadacycline Efficacy against Streptococcus Agalactiae Isolated in China: Correlation between Resistance and Virulence Gene and Biofilm Formation" was published in 2022. Journal: Comput Intell Neurosci.

**Figure 2:** The relationship among OMC, DOX, and MIN MIC distributions with ST10 (a) and ST17 (b) genotypes in *S. agalactiae.* Notes: OMC-omadacycline, DOX-doxycycline, MIN-minocycline, and TET-tetracycline.

**Table 1:** Comparison of in vitro antimicrobial activity of OMC and various common antibiotics against *S. agalactiae.*

Antibiotic	No of isolates (MIC/inhibition zone diameter)	MIC (mg/L)	Resistance rate (%)	MIC (Ug/Ml) breakpoint	N	Inhibition zone diameter (mm) a breakpoint	*N*
Total	162/*n*	—	—	—	—	—	—
Tigecycline	162	0.06–0.5	0	≤2	162	—	—
				4	0	—	—
				≥8	0	—	—
Doxycycline	162	0.25–22	22.2	≤0.25	12	—	—
				0.5	4	—	—
				≥1	110	—	—
Minocyclin	162	0.125–32	82.1	≤4	23	—	—
				8	4	—	—
				≥16	133	—	—
Eravacylcine	162	0.015–0.25	0	≤0.25	162	—	—
				0.5	0	—	—
				≥1	0	—	—
Omadacycline	162	0.25–0.5	13.6	≤0.25	68	—	—
				0.5	72	—	—
				≥1	22	—	—
Radezolind	162	0.03–1	0	≤2	162	—	—
				4	--	—	—
				≥8	--	—	—
Erytromycin	136/25	≤0.06–16	46.3/88.0	≤0.25	66	≥23	1
				0.5	7	14–22	2
				≥1	63	≤13	22
Solithromycin	142	0.015–2	54.2	≤0.25	21	—	—
				0.5	38	—	—
				≥1	77	—	—
Telavancin	139	0.06–2	—	≤0.12	24	—	—
				—	—	—	—
				—	—	—	—
Cefprozil	142	0.004–2	0	≤2	43	—	—
				4	0	—	—
				≥8	0	—	—
Tetracycline	162	—	—	≤1		—	—
				2		—	—
				≥4		—	—
Clindamycin	16	—	81.2	—	—	≥19	2
				—	—	16–18	1
				—	—	≤15	13
Chloramphenicol	39	—	15.4	—	—	≥21	11
				—	—	18–20	22
				—	—	≤17	6
Levofloxacin	16	—	25.0	—	—	≥17	8
				—	—	14–16	4
				—	—	≤13	4

Notes: OMC-omadacycline, DOX-doxycycline,, MIN-minocycline, and TET-tetracycline.

**Table 2:** Drug resistance rate of D-test against *S. agalactiae*.

Antibiotics	N	D-test		Drug resistance rate (%)
		D (+)	D (−)	
Omadacycline	162	15	147	90.74

**Table 3:** *In vitro* antimicrobial activity of OMC against *S. agalactiae* with TET-specific resistance genes.

TET resistance gene (S)	No.	ERAV MIC (mg/L)				OMC MIC (mg/L)				RADE MIC (mg/L)			
		≤0.25	0.5	≥1	Range	≤0.25	0.5	≥1	Range	≤2	4	≥8	Range
Tet (M)	71	71	0	0	0.008–0.25	32	28	8	0.25–1.00	—	—	—	—
Tet (O)	46	46	0	0	0.008–0.25	14	21	6	0.25–1.00	—	—	—	—
Tet (K)	44	44	0	0	0.008–0.25	14	26	6	0.25–1.00	—	—	—	—
Tet (M), tet (O)	7	7	0	0	0.008–0.25	4	0	2	0.125–1.00	—	—	—	—
Optra	13	—	—	—	—	—	—	—	—	13	0	0	0.06–0.25
None detected	9/149	9	0	0	0.015–0.25	4	2	3	0.25–1.00	149	0	0	0.03–0.25

**Table 4:** Relationships of OMC-resistant genes with biofilm formation in *S. agalactiae*.

OMC-resistant genes	Number and percentage of *Streptococcus agalactiae* (*N* = 136)											
	*N*	Strong		Medium		Weak		Negative		All positive		*P*-value
		*N*	%	*N*	%	*N*	%	*N*	%	*N*	%	
Erma (+)	0	0	0	0	0	0	0	0	0	0	0	0.145744203
Erma (−)	136	8	5.88	14	10.3	35	25.7	79	58.1	57	41.9	
Ermb (+)	98	7	7.14	11	11.2	29	29.6	51	52.0	47	48.0	0.122867448
Ermb (−)	38	1	2.63	3	7.89	7	18.4	27	71.5	11	28.9	
Ermc (+)	2	0	0	0	0	0	0	2	1.00	0	0	0.146326519
Ermc (−)	134	8	5.97	14	10.4	35	26.1	77	57.5	57	42.5	
Optra (+)	13	2	15.4	2	15.4	2	15.4	7	53.8	6	46.1	0.863018713
Optra (−)	126	6	4.76	12	9.52	35	27.8	73	57.9	53	42.1	
Cfr (+)	0	0	0	0	0	0	0	0	0	0	0	0.145744203
Cfr (−)	136	8	5.88	14	10.3	35	25.7	79	58.1	57	41.9	
Cfrb (+)	0	0	0	0	0	0	0	0	0	0	0	0.145744203
Cfrb (−)	136	8	5.88	14	10.3	35	25.7	79	58.1	57	41.9	
Msra (+)	0	0	0	0	0	0	0	0	0	0	0	0.145744203
Msra (−)	136	8	5.88	14	10.3	35	25.7	79	58.1	57	41.9	
Msrb (+)	0	0	0	0	0	0	0	0	0	0	0	0.145744203
Msrb (−)	136	8	5.88	14	10.3	35	25.7	79	58.1	57	41.9	
Mefae (+)	30	6	20.0	1	3.33	3	10.0	20	66.7	10	33.327	0.094142032
Mefae (−)	106	29	27.4	13	12.3	32	30.2	32	30.2	74	69.8	
Tetm (+)	61	5	8.20	3	4.92	16	26.2	37	60.7	24	39.3	0.74704373
Tetm (−)	75	3	4.00	11	14.7	19	25.3	42	56.0	33	44.0	
Teto (+)	46	2	4.34	7	15.2	12	26.1	25	54.3	21	45.7	0.504670116
Teto (−)	90	6	6.67	7	1.11	23	25.6	54	60.0	36	40.0	
Tetk (+)	27	1	3.70	2	7.40	10	37.0	14	51.9	13	48.1	0.696589923
Tetk (−)	109	7	6.42	12	11.0	25	22.9	65	59.6	44	40.4	

The article "Omadacycline Efficacy against Streptococcus Agalactiae Isolated in China: Correlation between Resistance and Virulence Gene and Biofilm Formation" was published in 2022. Journal: Comput Intell Neurosci.

**Table 5:** Relationships of OMC virulence genes with biofilm formation in *S. agalactiae*.

OMC virulence genes	*N*	Number and percentage of *Streptococcus agalactiae* (*N* = 136)										
		Strong		Medium		Weak		Negative		All positive		*P*-value
		*N*	%	*N*	%	*N*	%	*N*	%	*N*	%	
Bac (+)	136	8	5.88	14	10.3	35	25.7	79	58.1	57	41.9	0.145744203
Bac (−)	0	0	0	0	0	0	0	0	0	0	0	
Bca (+)	132	8	6.06	10	7.58	35	26.52	79	59.85	53	40.15	0.192189367
Bca (−)	4	0	0	4	1	0	0	0	0	4	1	
Fbsa (+)	53	8	15.1	12	22.6	26	49.1	7	13.2	46	86.8	0.073412483
Fbsa (−)	83	0	0	2	2.41	9	10.8	72	86.7	11	13.3	
Fbsb (+)	136	8	5.88	14	10.3	35	25.7	79	58.1	57	41.9	0.145744203
Fbsb (−)	0	0	0	0	0	0	0	0	0	0	0	
Cfb(+)	136	8	5.88	14	10.3	35	25.7	79	58.1	57	41.9	0.145744203
Cfb (−)	0	0	0	0	0	0	0	0	0	0	0	
Cfr (+)	136	8	5.88	14	10.3	35	25.7	79	58.1	57	41.9	0.145744203
Cfr (−)	0	0	0	0	0	0	0	0	0	0	0	
Hylb (+)	136	8	5.88	14	10.3	35	25.7	79	58.1	57	41.9	0.145744203
Hylb (−)	0	0	0	0	0	0	0	0	0	0	0	
Imb (+)	136	8	5.88	14	10.3	35	25.7	79	58.1	57	41.9	0.145744203
Imb (−)	0	0	0	0	0	0	0	0	0	0	0	
Cyle (+)	136	8	5.88	14	10.3	35	25.7	79	58.1	57	41.9	0.145744203
Cyle (−)	0	0	0	0	0	0	0	0	0	0	0	
Cpsa (+)	135	8	5.88	14	10.3	35	25.7	78	58.1	57	41.9	0.145744203
Cpsa (−)	1	0	0	0	0	0	0	1	100	0	0	
Scpb (+)	126	8	6.35	14	11.1	33	26.2	71	56.3	55	43.7	0.03921902
Scpb (−)	10	0	0	0	0	2	20	8	80	2	20	
Rib (+)	96	7	7.29	8	8.33	23	24.0	58	60.4	38	39.6	0.552661755
Rib (−)	40	1	2.50	6	15.0	12	30.0	21	52.5	19	47.5	
Cpsiii(+)	79	6	7.60	4	5.06	19	24.1	50	63.3	29	36.7	0.479252866
Cpsiii (−)	57	2	3.51	10	17.5	16	28.1	29	50.9	28	49.1	
Pi−1 (+)	0	0	0	0	0	0	0	0	0	0	0	0.145744203
Pi−1 (−)	136	8	5.88	14	10.3	35	25.7	79	58.1	57	41.9	
PI−2a (+)	0	0	0	0	0	0	0	0	0	0	0	0.145744203
PI−2a (−)	136	8	5.88	14	10.3	35	25.7	79	58.1	57	41.9	
PI−2b (+)	0	0	0	0	0	0	0	0	0	0	0	0.145744203
PI−2b (−)	136	8	5.88	14	10.3	35	25.7	79	58.1	57	41.9	

The article "Omadacycline Efficacy against Streptococcus Agalactiae Isolated in China: Correlation between Resistance and Virulence Gene and Biofilm Formation" was published in 2022. Journal: Comput Intell Neurosci.

## Data Availability

The datasets used and/or analyzed during the current study are available from the corresponding author on reasonable request.
